The article "Enhanced levels of Hsulf-1 interfere with heparin-binding growth factor signaling in pancreatic cancer" was published in 2005. Journal: Mol Cancer.

# Enhanced levels of Hsulf-1 interfere with heparin-binding growth factor signaling in pancreatic cancer

**DOI:** 10.1186/1476-4598-4-14

**Published:** 2005-04-07

**Authors:** Junsheng Li, Jörg Kleeff, Ivane Abiatari, Hany Kayed, Nathalia A Giese, Klaus Felix, Thomas Giese, Markus W Büchler, Helmut Friess

**Affiliations:** 1 Department of General Surgery, University of Heidelberg, Heidelberg, Germany; 2 Department of General Surgery, Zhong-Da Hospital, Southeast University, Nanjing, China; 3 Institute of Immunology, University of Heidelberg, Heidelberg, Germany

**Keywords:** pancreatic cancer, growth factors, sulfatase, proteoglycans

## Abstract

Hsulf-1 is a newly identified enzyme, which has the ability to decrease the growth of hepatocellular, ovarian, and head and neck squamous cell carcinoma cells by interfering with heparin-binding growth factor signaling. Since pancreatic cancers over-express a number of heparin-binding growth factors and their receptors, the expression and function of this enzyme in pancreatic cancer was analyzed.

**Results:**

Pancreatic cancer samples expressed significantly (22.5-fold) increased Hsulf-1 mRNA levels compared to normal controls, and Hsulf-1 mRNA was localized in the cancer cells themselves as well as in peritumoral fibroblasts. 4 out of 8 examined pancreatic cancer cell lines expressed Hsulf-1, whereas its expression was below the level of detection in the other cell lines. Stable transfection of the Hsulf-1 negative Panc-1 pancreatic cancer cell line with a full length Hsulf-1 expression vector resulted in increased sulfatase activity and decreased cell-surface heparan-sulfate proteoglycan (HSPG) sulfation. Hsulf-1 expression reduced both anchorage-dependent and -independent cell growth and decreased FGF-2 mediated cell growth and invasion in this cell line.

**Conclusion:**

High expression of Hsulf-1 occurs in the stromal elements as well as in the tumor cells in pancreatic cancer and interferes with heparin-binding growth factor signaling.

## Introduction

Pancreatic cancer is one of the most aggressive human malignancies with an overall five-year survival rate of less then 5% [1]. Although the reasons for the aggressive growth behavior of pancreatic cancer are not completely understood, recent molecular biological studies have revealed several factors that are involved in the pathogenesis of pancreatic cancer. These include genetic changes, such as k-ras, p53, p16, and Smad4 mutations [2], as well as epigenetic alterations, such as overexpression of a number of growth factors and their receptors [3,4].

Membrane-associated heparin-sulfate proteoglycans (HSPGs) are thought to play an important role in many aspects of cellular physiology including growth factor signaling. HSPGs are required for the optimal activity of heparin-binding growth factors, such as for example fibroblast growth factors (FGFs) [5,6]. One member of the HSPG family, glypican-1 is over-expressed in pancreatic cancer and influences heparin binding growth factor signaling in this disease [7,8]. The heparan-sulfate (HS) chains of HSPGs seem to interact with the ligands (e.g. FGF-2) and high-affinity FGF-receptors, to increase ligand-receptor binding and signaling [9]. The enzyme Hsulf-1 is a recently identified human sulfatase, which exhibits arylsulfatase activity [10]. Hsulf-1 expression is down-regulated in ovarian cancers, and lost in a proportion of liver cancers [11,12]. Absence or low levels of Hsulf-1 in hepatocellular, ovarian, and head and neck squamous cell carcinoma cell lines were associated with up-regulation of heparin-binding growth factor signaling [11-13]. Since HSPGs such as glypican-1 play an important role in pancreatic cancer and since Hsulf-1 can influence the sulfation state and the biological function of HSPGs, the expression and functional role of Hsulf-1 was analyzed in pancreatic cancer.

The article "Enhanced levels of Hsulf-1 interfere with heparin-binding growth factor signaling in pancreatic cancer" was published in 2005. Journal: Mol Cancer.

## Results

### Hsulf-1 mRNA expression in pancreatic tissues

Utilizing DNA arrays the expression of nine sulfatase family members in pancreatic cancer, pancreatic cancer metastasis, chronic pancreatitis and the normal pancreas was screened. This analysis revealed that Hsulf-1 was significantly over-expressed in pancreatic cancer and chronic pancreatitis compared to normal pancreatic tissues. Thus, Hsulf-1 mRNA expression levels were increased 9.1-fold in primary pancreatic cancer, 4.5-fold in pancreatic cancer metastasis, and 3.4-fold in CP tissues compared to normal pancreatic tissues. In contrast, there were only minor or no changes in the mRNA levels of the other members of the sulfatase family (Table 1). In order to better quantify Hsulf-1 expression quantitative RT-PCR was carried out in normal pancreatic tissue samples (n = 19), chronic pancreatitis (n = 22) and pancreatic cancer tissue samples (n = 31). The samples from normal tissues had a mean (+/- SEM) number of Hsulf-1 transcripts/μl of 114 ± 23, while Hsulf-1 mRNA levels increased in both chronic pancreatitis and pancreatic cancer, with mean (+/- SEM) transcripts levels of 2054 ± 911 in chronic pancreatitis and 2566 ± 420 in pancreatic cancer. 10 of 22 (45%) CP and 22 of 31 (71%) pancreatic cancer tissue samples displayed higher copy numbers of Hsulf-1 mRNA than the highest Hsulf-1 mRNA level observed in normal pancreatic tissue samples (Figure 1).

**Table 1:** Expression of different sulfatases in normal pancreas (No), chronic pancreatitis (CP), primary pancreatic cancer (CA) and pancreatic cancer metastasis (Mx) tissues as determined by DNA array analysis.

	**Fold change**		
	**Ca vs No**	**Mx vs No**	**CP vs No**

**hSulf-1**	**9.1**	**4.5**	**3.4**
**Arylsulfatase A**	0.6	0.8	0.9
**Arylsulfatase B**	1.8	1.6	1.8
**Arylsulfatase C**	1.6	1.8	1.6
**Arylsulfatase D**	0.5	0.2	0.8
**Arylsulfatase E**	0.5	0.6	0.7
**galactosamine (N-acetyl)-6-sulfate sulfatase**	0.8	0.8	0.9
**glucosamine (N-acetyl)-6-sulfatase**	2.5	2.2	1.6
**iduronate 2-sulfatase**	1.0	1.2	1.0

The article "Enhanced levels of Hsulf-1 interfere with heparin-binding growth factor signaling in pancreatic cancer" was published in 2005. Journal: Mol Cancer.

**Figure 1:** **Expression of Hsulf-1 mRNA in pancreatic tissues and cell lines **Quantification of Hsuf-1 mRNA levels in the normal pancreas, chronic pancreatitis (CP), pancreatic cancer tissues (PC), by real time QRT-PCR as described in the *Material and Methods *section. Values are normalized to housekeeping genes (cyclophilin B and HRPT), and presented as single values and mean (horizontal line).

### Localization of Hsulf-1 in pancreatic tissues

To identify the local expression pattern of Hsulf-1 in the normal pancreas, chronic pancreatitis and pancreatic cancer tissues, *in situ *hybridization analysis was carried out. Weak Hsulf-1 mRNA expression was observed in the acini of normal and chronic pancreatitis tissues. Hsulf-1 mRNA was localized in the smooth muscle cells and the endothelium of blood vessels, as well as in fibroblasts of the connective tissue (Figure 2 A–C). In addition, Hsulf-1 mRNA expression was present in tubular complexes of chronic pancreatitis tissues (Figure 2 D). In pancreatic cancer tissues, Hsulf-1 mRNA was mainly expressed in tubular complexes (Figure 2 E), in the cancer cells themselves (Figure 2 F, G) as well as in fibroblasts of the connective tissue (Figure 2 F).

**Figure 2:** **Expression and localization of Hsulf-1 mRNA in pancreatic tissues **In situ hybridization was performed as described in *Material and Methods *section. Hsulf-1 localization in: normal pancreatic acini (**A**); blood vessels (**B**), nerves (**C**), and tubular complexes (**D**) of CP; tubular complexes (**E**), cancer cells (**F**) of pancreatic cancer. Note the staining in the control section probed with the antisense riboprobe **(G)**, compared with absent staining in the sense-probed section (**H**).

### Hsulf-1 expression in pancreatic cancer cell lines

QRT-PCR analysis was carried out in 8 cultured pancreatic cancer cell lines. This analysis revealed relatively high expression of Hsulf-1 mRNA in Su-8686 and moderate expression in T3M4, Colo-357, and BxPc-3 pancreatic cancer cell lines. In the other cell lines, Hsulf-1 expression was below the detection level (Figure 3 A). Panc-1 pancreatic cancer cells were selected for Hsulf-1 transfection, since Hsulf-1 expression was below the level of detection in this cell line. To confirm successful transfection of Panc-1 cells with the full-length Hsulf-1 construct, Northern blot analysis was carried out using a Hsulf-1 antisense riboprobe. A total of number 36 clones were screened, of which 10 clones clearly expressed Hsulf-1 mRNA. Two Hsulf-1 positive clones (sulf-26 and sulf-38) were selected for use in further experiments and compared to empty vector-transfected (EV) and non transfected wild type (WT) Panc-1 cells (Figure 3 B). To confirm the expression of Hsulf-1 in the positive clones on the protein level, immunoblotting was performed. Since the Hsulf-1 expression plasmid contained a c-myc tag [10], it was possible to detect the expression of the Hsulf-1-myc fusion protein in the selected clones by immunoblot analysis with an anti-c-myc antibody (Figure 3 C). To determine the activity of the expressed sulfatase, cellular extracts prepared from both control (wild type and empty vector) and transfected clones (sulf-26, sulf-38) were analyzed. 4-Methylumbelliferyl-sulfate, which represents a substrate for a variety of sulfatases, including cellular steroid sulfatases, was used as the substrate for sulfatase activity. Upon transfection, sulfatase activity was most prominently increased in clone sulf-38 (Figure 3 D). However, since this assay could not differentiate between different sulfatases, high sulfatase activity was also observed in the control cells. Therefore, to further confirm successful transfection and increased Hsulf-1 activity, immunofluorescence with the 10E4 anti-HSPG monoclonal antibody, which recognizes N-sulfated glucosamine-containing HSPGs, was carried out. Prominent staining of the cell membrane was observed in both wild type (Figure 4A) and empty vector Panc-1 cells (Figure 4 C). In contrast, markedly diminished staining of the cell membrane was observed in the two Hsulf-1 expressing clones (Figure 4 B, D), indicating that Hsulf-1 desulfates HSPGs at the cell surface.

The article "Enhanced levels of Hsulf-1 interfere with heparin-binding growth factor signaling in pancreatic cancer" was published in 2005. Journal: Mol Cancer.

**Figure 3:** **Expression of Hsulf-1 in pancreatic cancer cell lines (A) **Quantification of Hsulf-1 mRNA levels in pancreatic cancer cell lines by real time QRT-PCR as described in the *Materials and Methods *section. Values are normalized to housekeeping genes (cyclopilin B and HRPT), and presented as mean ± SD. **(B/C) **Panc-1 cells were stable transfected with a Hsulf-1 sense expression plasmid as described in the *Material and Methods *section. **(B) **Hsulf-1 sense RNA expression in Panc-1 cells was verified by Northern blot analysis using a radiolabeled Hsulf-1 antisense riboprobe. A sample Northern blot of 2 controls and 2 transfected clones is shown. **(C) **Expression of c-myc tagged Hsulf-1 (arrow) by immunoblot analysis as described in the *Materials and Methods *section. Equal loading of the protein samples was confirmed using anti-γ-tubulin antibodies. **(D) **Sulfatase activity was measured as described in *Material and Methods *section in control and positive transfected clones. Data are expressed as relative fluorescence and presented as mean ± SD.

**Figure 4:** **Hsulf-1 decreases the sulfation of cell surface HSPGs **Immunofluorescence was performed as described in *Material and Methods *section with a specific 10E4 anti-HSPG monoclonal antibody, which recognizes native heparan-sulfate containing the N-sulfated glucosamine moiety. WT **(A)**, EV **(C)**, Sulf-26 **(B)**, Sulf-38 **(D)**.

### Functional consequences of Hsulf-1 expression in Panc-1 pancreatic cancer cells

Next, the effects of Hsulf-1 expression on the growth of Panc-1 cells were assessed. Analysis of basal growth revealed that the 2 control clones displayed an average exponential doubling time of 50.3 ± 3.2 hours, which was significantly shorter compared to the 2 Hsulf-1 transfected clones (68.2 ± 4.3 hours) (Figure 5 A). To determine anchorage-independent growth rates, soft agar assays were carried out. The 2 control clones showed an average colony number of 223 as compared to 31 colonies for the Hsulf-1 transfected cells (Figure 5 B).

**Figure 5:** **Hsulf-1 expression decreases Panc-1 pancreatic cancer cell growth **(**A**) Basal cell growth as determined by the MTT assay. Data are expressed as mean ± SD of three independent experiments. Data are presented for control cells (WT, EV), as well as for Hsulf-1 transfected clones. (Sulf-26, Sulf-38). (**B**) Anchorage-independent cell growth for individual clones was measured by the soft agar assay as described in the *Material and Methods *section. Data are presented for controls and positive clones as indicated. Data are presented as mean ± SEM obtained from three independent experiments.

### Hsulf-1 decreases FGF-2 mediated cell proliferation and signaling in Panc-1 pancreatic cancer cells

It has been shown previously that a variety of growth factors such as FGF-2, EGF, HB-EGF, and IGF-1 are over expressed in pancreatic cancer and that they have the potential to act as mitogens for pancreatic cancer cell lines [3,4]. Therefore, we further investigated whether over-expression of Hsulf-1 could modulate the function of these growth factors in pancreatic cancer cells. Two Hsulf-1 transfected clones and two controls (wild type and empty vector) were selected to perform growth assays in the presence or absence of different doses of the indicated growth factors. Hsulf-1 expression significantly attenuated FGF-2 (50 ng/ml) induced cell growth by around 50%, from +28.0 ± 3.8% in controls to +14.4 ± 1.0 % in Hsulf-1 clones (Figure 6). In contrast, there was no difference in the response towards IGF-1, EGF or HB-EGF in the control versus Hsulf-1 expressing cells. Since Hsulf-1 expression reduced FGF-2 but not EGF or HB-EGF induced cell proliferation, next we sought to investigate whether Hsulf-1 expression would influence FGF-2 and EGF/HB-EGF downstream signaling. EGFR phosphorylation was not changed in response to EGF or HB-EGF in Hsulf-1 expressing clones compared to controls (Figure 7 A). In addition, there was also no difference of EGF and HB-EGF induced MAPK phosphorylation between control cells and positive clones (Figure 7 A). In contrast, control cells showed increased MAPK phosphorylation after FGF-2 stimulation, while this FGF-2 induced phosphorylation was markedly attenuated in Hsulf-1 transfected cells (Figure 7 B). Next, the basal and FGF-2 induced invasion capacity of tumor cells was analyzed. This analysis revealed a significant reduction in the invasiveness of FGF-2 exposed Hsulf-1 expressing cells compared to Hsulf-1 negative clones. As demonstrated in Figure 7C, FGF-2 (10 μg/ml) significantly stimulated the invasion of the control cells by +83.4 ± 24.2% after 24 h of incubation. In contrast, the invasion ability of Hsulf-1 positive cells was significantly less stimulated (+27.4 ± 35.5%) by exposure to FGF-2 (Figure 7 C).

The article "Enhanced levels of Hsulf-1 interfere with heparin-binding growth factor signaling in pancreatic cancer" was published in 2005. Journal: Mol Cancer.

**Figure 6:** **Effects of Hsulf-1 expression on growth factor induced proliferation**. Clones were cultured in 1% FBS medium and incubated with increasing concentrations of the indicated growth factors for 72 h. Cell growth was measured by the MTT assay. Percent growth stimulation was determined by comparison with control cell growth. Values shown are the mean ± SEM obtained from three independent experiments.

**Figure 7:** **(A-B). Effects of Hsulf-1 on EGF/HB-EGF and FGF-2 induced receptor phosphorylation and MAPK phosphorylation. **Panc-1 pancreatic cancer cells were cultured in 1% FBS medium overnight and then incubated with 10 μg/ml of the indicated growth factors for 10 min. Phosphorylation of MAP kinase and receptor phosphorylation (EGFR) was determined by immunoblotting with antibodies specific for phospho-p44/42 MAPK and phospho-EGFR. Equal loading was determined by re-blotting the membranes with an γ-tubulin antibody. The figure is representative of three independent experiments. **(C) Hsulf-1 attenuates FGF-2 stimulated invasion. **An *in vitro *cell invasion assay was performed using 8 μM filters coated with Matrigel as described in the *Material and Methods *section. Panc-1 cells (1.25 × 10^5^) were seeded onto the filters in 1% serum overnight, and then treated as indicated for 24 h. The values shown are the mean ± SEM obtained from three independent experiments.

The article "Enhanced levels of Hsulf-1 interfere with heparin-binding growth factor signaling in pancreatic cancer" was published in 2005. Journal: Mol Cancer.

### Effects of Hsulf-1 expression on chemosensitivity

Pancreatic cancers exhibit variable degrees of chemotherapy resistance. To determine whether Hsulf-1 expression might influence the sensitivity of Panc-1 cells to chemotherapeutic agents, cells were treated with gemcitabine, 5-FU, or actinomycin-D and the GI50 concentration was calculated. The GI50 concentration of gemcitabine in the Panc-1 WT control cells was 3.9 nM, and in EV Panc-1 cells approximately 50 nM. Interestingly Hsulf-1 expressing cells exhibited GI50 values of more than 100 nM (Figure 8). In contrast no significant changes were observed in the sensitivity of Hsulf-1 positive clones and control cells towards 5-FU and actinomycin-D.

**Figure 8:** **Effects of Hsulf-1 on the sensitivity towards chemotherapeutic agents**. Panc-1 cells were cultured in complete medium and incubated in the absence (control) or presence of increasing concentrations of the indicated drugs for 48 h. Cell growth was measured by the MTT assay. Percent growth inhibition was determined by comparison with control cell growth. Values shown are the mean ± SEM obtained from three independent experiments.

## Discussion

Sulfatases are a family of enzymes that catalyse the hydrolysis of sulfate ester bonds from a wide variety of compounds. They are classified into arylsulfatases and nonarysulfatases according to their ability to hydrolyse the sulfate ester bonds of aromatic compounds such as p-nitrocatechol sulfate and 4-methylumbelliferyl sulfate [14]. Hsulf-1 is a newly identified member of the sulfatase family, which exhibits arysulfatase activity and removes sulfate from the C-6 position of glucosamine within the specific sub regions of intact heparin [10]. In the present study a significant up-regulation of Hsulf-1 in primary pancreatic cancer, pancreatic metastasis and CP compared to normal pancreatic tissues was demonstrated, whereas there was no significant difference in the expression of other members of the sulfatase family in these tissues. This indicates that Hsulf-1 might play a specific role in the pathogenesis and evolution of CP and pancreatic cancer. Normal pancreatic tissues are composed mainly of a homogenous population of acinar cells (and a low percentage of ductal and islet cells), whereas both CP and pancreatic cancer tissues contain a variable amount of desmoplastic areas, inflammatory cells, degenerating acini, tubular complexes (and cancer cells). Thus, the observed wide range of expression of Hsulf-1 mRNA in both CP and pancreatic cancer tissues is most likely due to the different individual composition of these tissues. To confirm this hypothesis, *in situ *hybridization was utilized to localize Hsulf-1 mRNA expression in normal, CP and pancreatic cancer tissues. This analysis demonstrated that Hsulf-1 mRNA expression was weakly present in normal acinar cells, and at high levels in the endothelium and smooth muscle cells of blood vessels, as well as in fibroblasts and tubular complexes in CP tissues and additionally in the malignant cells in pancreatic cancer tissues.

The article "Enhanced levels of Hsulf-1 interfere with heparin-binding growth factor signaling in pancreatic cancer" was published in 2005. Journal: Mol Cancer.

The observed increased levels of Hsulf-1 in pancreatic cancer tissues seem to be in contrast to the down-regulation of Hsulf-1 in HCC and ovarian tumors [11,12]. However, while in ovarian cancer markedly diminished levels were observed in approximately 75% of the cases [11], the percentage was much smaller in HCCs (30%) [12], suggesting that reduced Hsulf-1 expression is not universally observed in all tumor types. It has been hypothesized that enhanced expression of Hsulf-1 is related to c-myc amplification in HCCs [12]. It could be speculated that also in pancreatic cancer high Hsulf-1 levels are related to c-myc amplification [15], at least in a subset of tumors. Another interesting aspect is the generally low Hsulf-1 expression level in cultured cancer cell lines. Thus, Hsulf-1 expression is absent in 71% of ovarian cancer cell lines [11], in 82% of HCC cell lines [12], and in 50% of pancreatic cancer cell lines (present study).

To evaluate the functional importance of Hsulf-1 in pancreatic cancer cells, Panc-1 cells, which do not express Hsulf-1 at detectable levels, were stably transfected with a Hsulf-1 expression vector. Over-expression of Hsulf-1 in Panc-1 cells resulted in reduced anchorage-dependent and -independent cell growth, suggesting an important growth regulatory role of this gene in pancreatic cancer. These tumors are characterized by enhanced expression of a variety of growth factors and their receptors, which have the capacity to influence different cellular functions, such as cell proliferation, migration and angiogenesis [3,4]. Some of these growth factors are heparin-binding growth factors, such as FGFs, VEGF and HB-EGF. We hypothesized that Hsulf-1 expression would attenuate the effects of these growth factors by desulfation of HSPGs resulting in a growth disadvantage as suggested for other tumors [11-13]. FGF-2 stimulated cell proliferation was attenuated by the expression of Hsulf-1. Nonetheless, FGF-2 still induced growth in Hsulf-1 expressing cells, but to a lesser extent compared with control cells. It is conceivable that the HSPG/FGF receptor complex can facilitate FGF-2 signaling, but may not be strictly required for binding of FGF-2 to its receptor; it only increases the affinity of the FGF-2/FGF receptor interaction to a certain degree. Hsulf-1 expression in Panc-1 cells also partially blocked FGF-2 induced MAPK phosphorylation and invasion, further supporting the hypothesis that Hsulf-1 interferes with FGF-2 signaling in pancreatic cancer cells. In contrast, no difference between Hsulf-1 expressing and control cells was observed upon stimulation with HB-EGF – another heparin-binding growth factor- as well as EGF and IGF-1 suggesting that these growth factors and their receptors do not require sulfated HSPGs for effective signaling. The observation that Hsulf-1 expression does not interfere with HB-EGF signaling in pancreatic cancer cells is in contrast to recent studies in ovarian cancer cells [11], suggesting cell type specific differences.

The article "Enhanced levels of Hsulf-1 interfere with heparin-binding growth factor signaling in pancreatic cancer" was published in 2005. Journal: Mol Cancer.

Previously, it has been shown that Hsulf-1 expression enhances cisplatin-induced apoptosis in HCC cell lines [12]. In the present study, we did not observe increased sensitivity towards chemotherapeutic agents in Hsulf-1 expressing versus control cells. In contrast, Hsulf-1 expressing Panc-1 cells were more resistant to gemcitabine than the control cells, thereby suggesting that Hsulf-1 over-expression might confer increased chemoresistance to pancreatic cancer cells and thus provide them with a growth advantage. However, the reason behind this effect is currently not known and requires further analysis.

In conclusion, Hsulf-1 is up-regulated in pancreatic cancer and chronic pancreatitis compared to normal pancreatic tissues, mainly due to over-expression in the desmoplastic and cancerous tissue elements. Expression of Hsulf-1 in Panc-1 cells negatively influences growth and invasion by attenuating FGF-2 signaling, suggesting that Hsulf-1 plays a specific role in the pathogenesis of pancreatic cancer. Further experimental approaches, especially *in vivo *studies, will help to assess in more detail the role of this enzyme in human pancreatic cancer.

## Materials and methods

### Materials

DMEM, trypsin-EDTA, and penicillin-streptomycin were purchased from Invitrogen (Mannheim, Germany); FBS from PAN Biotech (Aidenbach, Germany); Gene screen hybridization transfer membranes from PerkinElmer Life Science (Boston, MA, USA); ^32^P CTP from Amersham Pharmacia Biotech (Freiburg, Germany); Lipofectamine reagent™ and TRIzol Reagent from Invitrogen (Karlsruhe, Germany); RiboMAX™ Large Scale RNA production system, antibiotic G-418 sulfate from Promega (Mannheim, Gemany); Gemcitabine-Hydrochloride from Lilly (Eli Lilly and Company Limited, Hampshire, UK); Recombinant human FGF-2, Recombinant human IGF-1, Recombinant human HB-EGF from R&D systems (Wiesbaden-Nordenstadt, Germany); p-EGFR (Tyr 1173) antibody from Santa Cruz Biotechnology (Santa Cruz, CA, USA), p-P44/42 MAPK (Thr202/Tyr204) antibodies from Cell Signaling Technology (Frankfurt, Germany); EGF from Upstate Biotechnology (Hamburg, Germany); monoclonal anti-Heparan sulfate (10-E4 epitope) from Seikagaju Corporation (Tokyo, Japan); Labeled goat anti-mouse IgM antibodies from Molecular Probes (Leiden, Netherlands); Anti-c-Myc antibody from Invitrogen (Karlsruhe, Germany); Anti-goat IgG HRP- linked antibodies, anti-mouse IgG HRP- linked antibodies, anti-rabbit IgG HRP- linked antibodies and ECL immunoblotting detection reagents from Amersham Biosciences (Freiburg, Germany); complete mini-EDTA-free protease inhibitor cocktail tablets from Roche (Mannheim, Germany); DIFCO Noble agar from DIFCO Laboratories (Detroit, MI,) All other reagents were from Sigma (Munich, Germany).

The article "Enhanced levels of Hsulf-1 interfere with heparin-binding growth factor signaling in pancreatic cancer" was published in 2005. Journal: Mol Cancer.

### DNA array

The GeneChip^® ^HG-U95Av2 array used in this study was fabricated by Affymetrix Inc. (Santa Clara, CA). Poly (A)^+ ^RNA isolation, cDNA synthesis, cRNA in vitro transcription, product purification and fragmentation was performed as described [16,17]. Hybridization of the fragmented in vitro transcription product to oligonucleotide arrays was performed according to the manufacturer instructions (Affymetrix Inc.).

### Patients and tissues collection

31 pancreatic cancer samples were obtained from patients (median age 62.5 years; range, 41–78 years), who underwent pancreatic resections for pancreatic cancer at the University Hospitals of Berne (Switzerland) and Heidelberg (Germany). 22 chronic pancreatitis samples were obtained from patients who underwent resection for chronic pancreatitis (median age 44 years range 22–66 years). 19 normal human pancreatic tissue samples were obtained from previously healthy individuals through an organ donor program (median age 45 years range 20–74 years). Immediately upon surgical removal, tissue samples were either snap-frozen in liquid nitrogen and then maintained at -80°C until use (for RNA extraction) or fixed in 5% formalin and embedded in paraffin after 24 h. All studies were approved by the Ethics Committees of the University of Heidelberg, and the University of Bern. Written informed consent was obtained from all patients.

### Cell culture

Pancreatic cancer cell lines were routinely grown in DMEM medium (Panc-1 and Mia-PaCa-2) or RPMI medium (Aspc-1, BxPc-3, Capan-1, Colo-357, SU-8686 and T3M4) supplemented with 10% fetal calf serum (FCS), 100 U/ml penicillin, and100 μg/ml streptomycin (complete medium). Cells were maintained at 37°C in a humid chamber with 5% CO_2 _and 95% air atmosphere.

The article "Enhanced levels of Hsulf-1 interfere with heparin-binding growth factor signaling in pancreatic cancer" was published in 2005. Journal: Mol Cancer.

### Real-time quantitative polymerase chain reaction (QRT-PCR)

All reagents and equipment for mRNA and cDNA preparation were purchased from Roche (Roche Applied Science, Mannheim, Germany). mRNA was prepared by automated isolation using the MagNA Pure LC instrument and isolation Kit I (for cells) and Kit II (for tissues). RNA was reverse transcribed into cDNA using the 1^st ^Strand cDNA Synthesis Kit for RT-PCR (AMV) according to the manufacturer's instructions. QRT-PCR was performed with the Light Cycler Fast Start DNA SYBR Green kit as described previously [18]. The number of specific transcripts was normalized to housekeeping genes (cyclophilin B and hypoxanthine guanine phosphoribosyltransferase, HPRT), and presented as adjusted transcripts / μl cDNA. All primers were obtained from Search-LC (Heidelberg, Germany).

### In situ hybridization

Specific human Hsulf-1 riboprobes were generated by reverse-transcription polymerase chain reaction using the following primer pairs: Hsulf-1: sense, 5'-ACT GTA CCA ATC GGC CAG AG-3'; antisense, 5'-CCT CCT TGA ATG GGT GAA GA -3'. The resulting polymerase chain reaction products were subcloned into the pGEM-T easy vector (Promega GmbH, Mannheim, Germany) containing promoters for DNA-dependent SP6 and T7 RNA polymerases. The authenticity of the subcloned Hsulf-1 fragment was confirmed by sequencing (Qiagen GmbH, Hilden, Germany). Plasmids were linearized using SpeI and NcoI restriction enzymes. T7 and SP6 RNA polymerases were used to construct sense and antisense complementary RNA riboprobes. Biotin complementary RNA labeling was performed using the biotin RNA labeling kit according to the manufacturer's instructions (Roche Diagnostics, Mannheim, Germany). Tissue sections (3 μm) were deparaffinized, rehydrated with 1× phosphate-buffered saline, and incubated in 0.2 M/L HCl for 20 minutes at room temperature. After rinsing the slides in 2× standard saline citrate, sections were treated with proteinase K (Roche Diagnostics) at a concentration of 25 μg/ml for 15 minutes at 37°C. After postfixation with 4% paraformaldehyde in phosphate-buffered saline for 5 minutes and washing in 2× standard saline citrate, samples were acetylated in 2.5% acetic anhydride and 1.5% triethanolamine for 10 minutes. Subsequently, sections were prehybridized at 78°C for 2 hours in 50% formamide, 4× standard saline citrate, 2× Denhardt's reagent, and 250 μg RNA/ml. Hybridization was performed overnight at 78°C in 50% formamide, 4× standard saline citrate, 2× Denhardt's reagent, 500 μg RNA/ml, and 10% dextran sulfate. The final concentration of the biotin-labeled probes was 0.8 ng/μl. After hybridization, excess probe was removed by washing the slides 3 times in Dako stringent wash solution (Dako) at 78°C for 15 minutes. The samples were then incubated with streptavidin alkaline phosphatase conjugate (Dako) for 30 minutes at room temperature. For the color reaction, 5-bromo-4-chloro-3-indolyl phosphate/nitroblue tetrazolium substrate (Dako) was used.

The article "Enhanced levels of Hsulf-1 interfere with heparin-binding growth factor signaling in pancreatic cancer" was published in 2005. Journal: Mol Cancer.

### Stable transfection

The Hsulf-1 expression plasmid (pcDNA 3.1/myc-His) [10] was a kindly provided by S.D. Rosen (University of California, San Francisco). Panc-1 pancreatic cancer cells were stably transfected with the Hsulf-1 plasmid and with the empty control vector using the lipofectamine reagent [7,8]. Briefly, after reaching confluence, cells were split 1:10 into selection medium (complete medium supplemented with 1200 μg/ml G418) and single clones were isolated after 2–4 weeks. After expansion, cells fromeach individual clone were screened for the expression of Hsulf-1 by Northern blot analysis. Parental Panc-1 pancreatic cancer cells were also transfected with an empty expression vector carrying the neomycin-resistance gene as a control. Positive clones were routinely grown in selection medium.

### RNA extraction and Northern Blot analysis

The pGEMT-easy vector containing the Hsulf-1 fragment was linearized with SpeI, and a ^32^P -labeled riboprobe was synthesized with the RiboMAX™ large scale RNA production system kit using T7 polymerase and ^32^P CTP. Total RNA was extracted by the single step-acid guanidinium thiocyanate phenol chloroform method [7,8]. RNA (15 μg/lane) was size fractionated on 1.2 % agarose/1.8 M formaldehyde gels. Gels were stained with ethidium bromide for verification of RNA integrity and loading equivalency. Fractionated RNA was transferred onto Genescreen membranes and cross linked by UV irradiation. Blots were then prehybridized for 12 h at 65°C in 50% formamide, 1% SDS, 5 × Denhardt's, 100 μg/ml salmon sperm DNA, 50 mM Na_2_PO4, pH 7.4, 10% dextran, 75 mM NaCl and 5 mM EDTA. Blots were then hybridized for 24 h at 65°C in the presence of ^32^P CTP labeled riboprobe, rinsed twice with 2 × SSC and washed twice with 0.2 × SSC/2%SDS at 65°C for 20 min, respectively. All blots were exposed at -80°C to Kodak BiomaxMS films with Kodak-intensifying screens.

### Immunoblot analysis

Cell culture monolayers were washed twice with ice-cold PBS and lysed with lysis buffer (50 mM Tris-HCl, 100 mM NaCl, 2 mM EDTA,1% SDS) containing one tablet of complete mini-EDTA-free protease inhibitor cocktail (in 10 ml buffer). Protein concentration was determined by the BCA protein assay (Pierce Chemical Co, Rockford, IL,). Cell lysates (30 μg/lane) were separated on SDS-polyacrylamide gels and electroblotted onto nitrocellulose membranes. Membranes were then incubated in blocking solution (5% nonfat- milk in 20 mM Tris-HCl, 150 mM NaCl, 0.1% Tween-20), followedby incubation with the indicated antibodies at 4°C overnight. The membranes were then washed in blocking solution and incubatedwith HRP-conjugated secondary antibodiesfor 1 hour at room temperature. Antibody detection was performedby an enhanced chemiluminescence reaction.

The article "Enhanced levels of Hsulf-1 interfere with heparin-binding growth factor signaling in pancreatic cancer" was published in 2005. Journal: Mol Cancer.

### Sulfatase assay

To assay sulfatase activity in whole cell extracts, cells were lysed in lysis buffer (10 mM HEPES, 150 mM NaCl, 1% NP-40, 10% glycerol, 1.0 mM PMSF, and 1 mM EGTA), and the lysates were incubated on ice for 10 minutes. 4-Methylumbelliferyl-sulfate was used as the substrate. Cell lysates with 100 μg protein were diluted with SIE (250 mmol/l sucrose, 3 mmol/L imidazole, 0.1% absolute ethanol, pH 7.4) to a total volume of 100 μl. One hundred μl of 1 μmol/l 4-methylumbelliferylsulfate was added to each tube, mixed, and incubated at 37°C for 12 hours. 2 ml of stop solution (50 mM glycine, 5 mM EDTA, pH 10.4) was then added and mixed, and released 4-methylumbelliferone was measured using a fluorometer (excitation wavelength 360 nm, emission wavelength 460 nm).

### Immunofluorescence assay

Cells were grown in complete medium overnight in 10-well chambers, washed with PBS, fixed with 4% formaldehyde/PBS for 20 min at room temperature (RT), incubated in ice-cold methanol for 5 min (RT) and subsequently in acetone for 2 min (RT). Cells were incubated overnight with an anti-mouse antibody that recognizes negative heparan sulfate that contains the N-sulfated glusamine residue (10E-4 mAb; 1:30 dilution) (Seikagaku Corporation Tokyo, Japan). Cells were then washed 3 times with PBS, incubated with Alexa Fluor labeled goat anti-mouse IgM antibodies (Molecular Probes, Leiden, Netherlands) for 1 hour at room temperature, washed with PBS and mounted with DAPI and anti-fading medium (Gel/mountTM, Abcam, Cambridgeshire, UK). Confocal microscopic analysis was performed using the Spectral Confocal Microscope Leica TCS SL (Leica Microsystems GmbH, Heidelberg, Germany).

### Proliferation assay

Anchorage-dependent cell growth was determined by the 3-(4,5-methylthiazol-2-yl)-2,5-diphenyltetrazolium bromide (MTT) colorimeric growth assay [7]. Briefly, 2,000 cells/well were plated in 96-well plates and cultured for up to 7 days. Each day cell growth was determined by adding MTT solution (50 μg /well) for 4 hours. Cellular MTT was solubilized withacidic isopropanol and optical density was measured at 570 nm. The doubling time was calculated for the exponential growth phase. To measure and calculate the GI_50 _of the chemotherapeutic agent (the concentration that causes 50% cell growth inhibition), graded concentrations of drugs were added to triplicate wells and GI_50 _was calculated using the formula 100 x (T-T_0_)/(C-T_0_) = 50, where T is the optical density of the test well after 48 hours period of exposure to drugs, T_0 _is the optical density at time zero, and C is the control optical density after 48 hours [19]. All experiments were performed in triplicate.

The article "Enhanced levels of Hsulf-1 interfere with heparin-binding growth factor signaling in pancreatic cancer" was published in 2005. Journal: Mol Cancer.

### Soft agar assay

Cells (1 × 10^3^/well) were suspended in 3 ml of 0.3% Difco Noble agar supplemented with complete culture medium. This suspension was layered over 1.5 ml of 0.5% agar-medium base layer in 12-well plates. After 14 days, cells were stained with MTT (400 μg/well) for 24 h and colonies larger than 0.05 mm were counted.

### Invasion assay

8 μm filters were coated with Matrigel and placed in chambers. Cells (1.25 × 10^4^) cells were cultured in DMEM medium containing 1% FBS overnight. FGF-2 was added to the top chambers. After a subsequent 24 h incubation at 37°C, non-invaded cells were scraped off, and the cells that migrated to the lower surface of the filter inserts were fixed with 25% acetic acid and 75% methanol for 10 min and stained with 1% Toluidine blue in 1% sodium borate solution. The invasion index was expressed as the ratio of the percent invasion of the treated cells over the percent invasion of the control cells.

### Statistical analysis

Results were expressed as mean ± SEM, unless indicated otherwise. For statistical analysis, the Student's t test was used. Significance was defined as *p *< 0.05.

## Competing interests

The author(s) declare that they have no competing interests.

## Authors' contributions

J.L, I.A, H.K carried out the in situ hybridization, immunoblotting, cell proliferation, invasion assays, and soft agar experiments. N.A.G. and T.G carried out the QRT-PCR analysis. J.K, M.W.B. and H.F. conceived the study and participated in its design and coordination. J.K. and K.F. drafted the manuscript. All authors read and approved the final version.
